# The Association between Emotional Stress, Sleep Disturbance, Depression, and Burning Mouth Syndrome

**DOI:** 10.1155/2021/5555316

**Published:** 2021-03-13

**Authors:** Fahimeh Rezazadeh, Farzane Farahmand, Hamidreza Hosseinpour, Reza Shahriarirad, Amirhasan Sabet Eghlidi

**Affiliations:** ^1^Department of Oral and Maxillofacial Medicine, Oral and Dental Diseases Research Center, School of Dentistry, Shiraz University of Medical Sciences, Shiraz, Iran; ^2^Student Research Committee, School of Dentistry, Shiraz University of Medical Sciences, Shiraz, Iran; ^3^Department of surgery, Shiraz laparoscopic research center, Shiraz University of Medical Sciences, Shiraz, Iran; ^4^Thoracic and Vascular Surgery Research Center, Shiraz University of Medical Sciences, Shiraz, Iran

## Abstract

**Introduction:**

Burning mouth syndrome (BMS) is one of the challenging clinical problems not only in its diagnosis and treatment but also its concurring mental impact. This study is aimed at determining the association between psychological factors, including emotional stress, depression, anxiety, and sleep pattern among BMS patients.

**Methods:**

In this cross-sectional study, 19 patients with idiopathic BMS were enrolled along with a control group equivalent in age and sex, but without BMS. Questionnaires used were the Visual Analog Scale (VAS), the Pittsburgh Sleep Quality Index (PSQI), and the Depression, Anxiety, and Stress Scale (DASS-21). Demographic information was also recorded and analyzed.

**Results:**

There was a significant correlation among the two groups of BMS and non-BMS patients regarding stress, depression, and sleep disorder. The average severity of the burning score was 8.31 among the patients. Furthermore, a significant correlation was observed among mental disorders and educational level and sex, but not with age. There was also no significant correlation among the severity of the burning score with sex, education, and mental disorder.

**Conclusion:**

BMS is significantly associated with psychological symptoms. This condition requires proper treatment and support because it can represent psychological or mental issues and/or have a significant effect on daily life.

## 1. Introduction

Burning mouth syndrome (BMS) is defined as a burning sensation in the normal oral mucosa without any laboratory and clinical findings associated with any medical or dental condition [1]. Middle-aged women are the most affected patients with a female to male ratio of 3 : 1 [2, 3]. Although actual global epidemiological data are limited, the prevalence of BMS is about 1 to 4% worldwide [3].

Various etiologies can lead to BMS, and there may be contributed to more than one factor, which makes patients see different medical specialists, including dentists, ENT specialties, and dermatologists [4]. The variety of etiological factors makes the diagnosis of BMS more challenging for healthcare providers. One of the first essential steps in patients with BMS is to rule out other dental causes and systematic medical conditions [5]. Although different research studies have tried to determine the exact characteristic findings and associated conditions, which lead to BMS, the correlation of factors such as depression, stress, and sleep disturbance has never been rigidly determined [6].

On the one hand, anxiety and depression are assumed as two common conditions playing a significant role in BMS [7]. On the other hand, it seems that pain catastrophizing is somehow more important than psychological disturbance and also sleep quality in these patients experiences [8]. However, researchs emonstrated the possibility of an association between poor sleep quality and oral burning in patients with BMS [9].

This study is aimed at describing the correlation of BMS and psychological variables, including anxiety and emotional stress, and to determine whether sleep disturbance and depression would play a critical role in characteristic symptoms of patients with BMS or not.

## 2. Methods and Materials

This cross-sectional study examines the rate of stress, anxiety, depression, and sleep disorders in patients with primary burning mouth syndrome who were referred to the Oral medicine Department of Shiraz Dental School from December 2019 to June 2020. Due to the low prevalence of this disease and the COVID-19 pandemic, which led to a decrease in patients referred to the clinic, we decided to select any number of patients with primary BMS referred to Shiraz Dental School for six months who fulfilled the inclusion criteria as the study population. All patients were informed about the voluntarily nature of participating in the study and were asked to fill out written informed consents. We used a convenience sampling method, in which if the person did not agree to the questionnaire or did not accept the terms of the study, the next person was replaced. The participants were grouped as either the case (patients with BMS) or control (healthy) group.

The inclusion criteria for the BMS group included the presence of pain lasting more than 6 months which continues throughout the day and without paroxysm and not following any unilateral nerve trajectory; chronic pain in the oral mucosa in the absence of hard and soft tissue lesions of any kind; and the absence of any abnormalities in laboratory findings, salivary flow rates, and Candidiasis detection tests [10]. A final diagnosis of BMS was confirmed by an oral medicine specialist after all other possible causes of oral complaints had been ruled out. The healthy group consisted of participants who visited our clinic and had no signs of oral mucosal lesions. The age limit for all participants was set as older than 18 years. Furthermore, those who were suffering from other systemic medical conditions, autoimmune diseases, and psychiatric problems and also patients who consumed any medication that affected sleep patterns or stress and anxiety were excluded from both groups. Age and sex were equalized between the case and control groups. According to these conditions, the sample size for each group was 19 people.

Data collection was carried out by a researcher who was blinded to the grouping of the patients. Demographic information (age, sex, and level of education) was recorded in both target and control groups. The severity of burning was determined using the Visual Analog Scale (VAS) and was divided into two categories: mild (0-5) and severe [6–10]. All participants were given the Pittsburgh Sleep Quality Index (PSQI) [11] to assess sleep quality and the Depression, Anxiety, and Stress Scale (DASS-21) questionnaire [12] to assess psychiatric factor disturbances. The present study was approved by the Medical Ethics Committee of the academy. (IR.SUMS.DENTAL.REC.1399.031).

Data analysis was performed by SPSS software version 21, and statistical methods of *t*-test, ANOVA, and Chi-square were used. Finally, the results were analyzed and confirmed by a psychiatrist. The significance threshold was set at 0.05.

## 3. Results

In this study, 19 patients were selected as the patient group and 19 people as the control group. The demographic features of the patients in our study are demonstrated in Table 1. There was no statistically significant difference between the two groups in terms of age (*P* = 0.312) or education (*P* = 0.732). The severity of burning was reported severe in 78.94% of patients (6 to 10 on the VAS scale) and the mean of VAS score was 8.31 among the patient group. In terms of stress, depression, and sleep disorders, a statistically significant increase was found in the patient group versus the control group (*P* = 0.001, 0.006, and 0.001, respectively). Interestingly, there was no significant association between BMS and anxiety (*P* > 0.05).

The relationship between the severity of burning and the demographic variables in our study was also evaluated in which the results are demonstrated in Table 2. The results of the statistical analysis did not show a significant relationship between the severity of burning and sex, level of education, and mental disorders (*P* > 0.05).

Table 3 demonstrates the correlation among mental disorders and age, sex, and educational level. Higher educational level (above diploma) was significantly associated with higher rate of psychological instabilities such as depression, stress, and anxiety (*P* = 0.001, 0.001, and 0.002, respectively); however, the association between educational level and sleep disturbance were not significant (*P* > 0.05). Also, the results of statistical analysis showed a significant relationship between sex and stress, depression, anxiety, and sleep disorders (*P* = 0.018, 0.004, 0.004, and 0.018, respectively). Apart from sleep problems, other disorders were more common in males relative to females. There was no significant relationship between age and stress, anxiety, depression, and sleep disorders in both groups (*P* > 0.05).

## 4. Discussion

Since BMS is a chronic disturbing disease with no efficient treatment, it can be expected that it can lead to negative emotional states. On the other hand, some studies have demonstrated that patients with psychological disorders can develop BMS [7]. Psychological abnormalities have been reported to be related to BMS in several studies [13–15] but the precise relationship between these factors and any predisposition to BMS remains unclear and the exact cause and effect in this regard is still a matter of debate. In this study, we aim to evaluate the association between oral symptoms of BMS and the psychological status of these patients.

The result of the current study shows a statistically significant increase in depression, stress, and sleep disorders among the BMS patients compared to the healthy volunteers. Therefore, based on our findings, psychological disorders seem to be associated with BMS. In accordance with our study, several previous studies have reported that 44% to 92% of patients with BMS have psychiatric disorders of which anxiety and depression are the most common [16–19]. The association of anxiety and depression with BMS and the improvement of this disease due to cognitive-behavioral therapies and antianxiety drugs indicate that mental illnesses may predispose patients to the development of BMS [20]. However, contrary to our findings, a number of studies have not shown a relationship between psychological disorders and BMS [21, 22]. The role and effect of psychological factors in BMS still require further investigation and individuals, especially healthcare workers should be aware of the risk of the concurrence of these two conditions to take necessary actions.

In our study, there was no significant correlation among BMS and anxiety among the patients. Nevertheless, Bakhtiari et al. [23] reported a significant difference in the level of anxiety in BMS patients versus healthy volunteers; however, this association was not observed in our study. Some studies emphasize that there is a relation between BMS and anxiety; however, there is still no clear cause-and-effect relationship between these two factors. The patient's history can help determine whether this feeling was before or after the behavior change.

Mental illnesses such as depression and anxiety play an important role in regulating the sensation of pain and are able to increase or decrease the neurotransmission of peripheral pain receptors and change the pain sensation and reduce the pain threshold of a person to receive a normal stimulus as a painful stimulus [19, 20]. In the present study, regarding the severity score for pain, an average VAS score of 8.31 was recorded and almost three-quarters of the patients (78.94%) had values of higher than 5, which is in the severe pain spectrum but without any significant association with any of our variables. However, in a study by Di Stasio et al. in Italy, an average VAS score of 6.22 in BMS patient was achieved which was significantly correlated with distress and depressive symptoms [24]. The insignificant in our study could be due to the small sample size or the disproportion of male to female ratio.

Regarding the relationship between sleep disorders and BMS, to the best of our knowledge, there was not found any similar study; however, some literature has shown that patients with chronic pain have poor sleep quality. The study of Almoznino et al. stated that 50% to 70% of patients with chronic pain have poor sleep quality compared to the control group [25]. In an Italian multicenter study, in agreement with the findings of other studies reported in the literature, they have found a prevalence of sleep disturbance in 79% of BMS patients that is in line with our result, in which we found sleep disturbance as a major complication of BMS with the incidence of 89.5% [26]. Lee et al. reported that BMS patients showed poor sleep quality, anxiety, and depression, as compared with the controls [8]. Sheng et al. reported that chronic pain can aggravate depression due to the stressful condition that they experience. Also, their results showed that more than 50% of patients with chronic pain suffer from depression [27]. All these studies highlight the relationship between oral burning, sleep, and mood.

The results of our study demonstrate a significant association between mental disorders with sex and education. Zeltzer et al. stated that the female sex, low level of education, celibacy, low income, old age, etc. are risk factors for anxiety [28]. However, the claim of the “protective effect” of education against depression has been challenged [29]. Contrary to these findings, the results of the current study indicate that people with higher education (above diploma) are significantly more prone to depression, stress, and anxiety (*P* < 0.05). Unlike previous studies, in the current study, no significant relationship was found between age (Table 3) and mental disorders and sleep disorders (*P* > 0.05).

Due to the fact that the rate of depression is higher among females than males, the relationship between the level of education and depression is complex and may vary based on sex [30, 31]. Unlike boys, the prevalence of depression among girls increases significantly through aging [32]. Contrary to the results of previous studies, although in the present study, a significant relationship was found between the incidence of mental illnesses such as stress, anxiety, and depression with sex (*P* < 0.05), but these disorders were more pronounced among men in our statistical group according to Table 3. Furthermore, a study by Naylor et al. in Iraqi and Afghan societies found that women with chronic pain reported higher rates of pain than men [33]. However, our study demonstrated no significant correlation between the severity of the burning of BMS patients and sex. Incompatibility of results can be due to the imbalance of male to female ratio in our study.

At the time of this study, due to the prevalence of the COVID-19 pandemic, the number of patients referred to Shiraz Dental School had strongly decreased and therefore only a limited number of patients were evaluated; However, it should be kept in mind that the opposed situation of the COVID-19 pandemic could also affect the mental health of the population [34–36]. Also, our population was mostly female patients which cause a sex bias among the results. It is recommended that a study with a larger sample size to be performed and that people who have psychological symptoms based on the information obtained from the questionnaires be examined by a psychiatrist to confirm the psychological disorder, which requires the formation of a team of at least one oral health specialist and psychiatrist to be stationed in one place and evaluate patients. Otherwise, due to the nonacceptance of most patients to see a psychiatrist, a large number of patients will be excluded from the study. Also, due to the limited access to hospital equipment, we were unable to evaluate the patients sleep disturbance based on polysomnography results, which could have documented solid proof of the effect of BMS on the patients sleep.

## 5. Conclusion

Based on the results of the present study, a statistically significant difference was observed between the two groups in terms of psychological symptoms. In order to help and elaborate on the role of psychological variables, investigate the interplay of particular cognitive and personality aspects, and evaluate the potential impact of life experiences, more research on BMS is required. Owing to the lack of available appropriate drugs and the lack of awareness from friends and family, patients with BMS suffer from distress and often frustration. This condition requires proper treatment and support because it can represent psychological or mental issues and/or have a significant effect on everyday life.

## Figures and Tables

**Table 1:** Investigation of age, sex, and level of education and mental disorders in two groups based on the patients reports.

Variables	Groups	Patient group *n* = 19	Control group *n* = 19	*P* value
Age (mean)		54.68	50.63	0.312

Sex (%)	Male	15.79	15.79	<0.001
	Female	81.24	81.24	

Education level (%)	Under diploma	31.6	36.8	0.732
	Above diploma	68.4	63.2	

Burning severity (Visual Analog Scale score)	0-5	21.05	—	—
	6-10	78.94	—	

Stress (%)	Yes	63.2	0	<0.001
	Mild	52.6	0	
	Moderate	10.5	0	
	No	36.8	100	

Anxiety (%)	Yes	57.9	21.1	0.05
	Mild	15.8	10.5	
	Moderate	42.1	10.5	
	No	42.1	78.9	

Depression (%)	Yes	63.2	21.1	0.006
	Mild	57.9	5.3	
	Moderate	10.5	10.5	
	No	36.8	78.9	

Sleep disorder (%)	Yes	89.5	31.6	<0.001
	No	10.5	68.4	

**Table 2:** Evaluation of the relationship between the severity of burning sensation based on the patients reports with sex, educational level, and mental disorders.

Variables	Groups	Severity of burning sensation		*P* value
		Mild *n* = 4	Severe *n* = 15	
Sex (%)	Male	18.8	81.2	0.53
	Female	33.3	66.7	
Education level (%)	Under diploma	50	50	0.071
	Above diploma	7.7	92.3	
Stress (%)	Yes^∗^	10.1	89.9	0.451
	No^∗^	37.5	62.5	
Anxiety (%)	Yes^∗^	8	92	0.269
	No^∗^	42.9	57.1	
Depression (%)	Yes^∗^	8	92	0.404
	No^∗^	51.7	42.9	
Sleep disorder (%)	Yes^∗^	23.5	76.5	1
	No^∗^	0	100	

**Table 3:** Evaluation of mental disorders based on age, sex, and educational level.

Mental disorder	Groups	Variables									
		Age (mean ± SD)	*P* value	Sex (%)				*P* value	Education level (%)		*P* value
				Male		Female			Under diploma	Above diploma	
				Case	Control	Case	Control				
Depression	Yes	56.18 ± 14.88	0.129	100	0	56.2	0	0.004	0	100	<0.001
	No	50.09 ± 9.31		0	100	43.8	100		85.7	14.3	
Stress	Yes	59.41 ± 13.7	0.018	100	0	56.2	0	0.018	0	100	<0.001
	No	49.53 ± 10.21		0	100	43.8	100		85.7	14.3	
Anxiety	Yes	56.13 ± 15.40	0.158	100	100	50	6.2	0.004	0	100	<0.001
	No	50.39 ± 9.21		0	0	50	93.8		75	25	
Sleep disorder	Yes	51.33 ± 9.13	0.595	33.3	0	100	37.5	0.018	35.3	64.7	1
	No	53.52 ± 13.94		66.7	100	0	62.5		0	100	

## Data Availability

SPSS data of the participant can be requested from the authors. Please write to the corresponding author if you are interested in such data.
